RETRACTED

# How do Institutional Investors Influence Corporate Governance under Legal Psychology

**DOI:** 10.1155/2022/5004309

**Published:** 2022-08-08

**Authors:** Sheng Qi

**Affiliations:** Law School, Henan University of Science and Technology, Luoyang 471000, China

## Abstract

In order to give full play to the role of field research of legal psychology institutional investors in promoting enterprise environmental governance, this article puts forward the research on how legal Psychology institutional investors affect the corporate governance environment. Taking the listed companies in the A-share heavy pollution industry of Shenzhen Stock Exchange from 2018 to 2021 as a sample, this article tests the impact and action mechanism of legal Psychology institutional investors' field research on corporate environmental governance. Hypothesis 1: the field research of legal Psychology institutional investors can promote the environmental governance of enterprises. Hypothesis 2: for enterprises with poor environmental information disclosure, the impact of field research of legal Psychology institutional investors on enterprise environmental governance is more obvious. Hypothesis 3: for enterprises with more concentrated distribution, the impact of field research of legal Psychology institutional investors on enterprise environmental governance is more obvious. Leadership power has the three attributes of management, social psychology, and law, and its essence is the socialization of legal psychology. Under the perspective of legal psychology, the psychological mechanism of leadership power is mainly manifested in three aspects: increasing the social distance, activating the approach system, and inducing the control illusion. The cumulative number of field investigations conducted by the enterprise in the current year +1 is adopted, and the logarithm is taken as the measurement index of the field investigation of legal Psychology institutional investors, which is expressed by Investigate. In the robustness test part, the virtual variables are set by whether the enterprise is investigated in the field in that year. The results show that in uncontrolled years and industries, the regression coefficients of legal Psychology institutional investor investigation and enterprise environmental protection capital investment are 0.0703 and 0.2416, respectively, which are significant at the level of 5%. After controlling the year and industry, the regression results show that the field investigation of legal Psychology institutional investors and enterprise environmental capital investment are still positive, significantly at the level of 5% and 1%, respectively. The environmental capital investment of enterprises with poor environmental information disclosure (0.479 and 1.161) is higher than that of enterprises with good environmental information disclosure (0.252 and 0.618), and the mean *t*-test maintains the significance level of 1%, indicating that the impact of field research on enterprise environmental governance is more obvious in enterprises with poor environmental information disclosure, which preliminarily verifies Hypothesis 2 of this article. Similarly, when the distribution of enterprises is more concentrated, the environmental capital investment of enterprises is 0.536 and 1.286, which is higher than that of enterprises with a more dispersed distribution (0.315 and 0.778) and maintains a significant level of 1%. The results show that obtaining environmental information is helpful for stakeholders to supervise enterprise environmental governance. Therefore, we should formulate and issue policies and regulations that require enterprises to disclose environmental information as soon as possible, improve the standards of environmental information disclosure, establish an enterprise environmental information disclosure platform, and improve the level and quality of environmental information disclosure.

RETRACTED

## 1. Introduction

Investment activities are the core part of the company's financial activities. Reasonable investment decisions are directly related to the value promotion and sustainable development of enterprises. The report of the 19th CPC National Congress clearly highlighted the importance of promoting effective investment and implementing the status of investment subject as well as deepening the reform of China's investment and financing system. Combing the government work reports over the years, it can be found that from 2017 to 2019, the words “effective investment” and “expanding investment” are the focus of continuous emphasis in the government work report. China will further deepen the reform of the financial market, reasonably expand effective investment, promote high-quality economic development, and constantly stimulate the vitality of social investment [1]. From the existing research, capital investment has always been the mainstream direction for scholars to study macro-economy. An accurate grasp of investment decision-making is related to the effective allocation of enterprise resources and sustainable operation and development.  Figure 1 shows the industrial chain of private equity investment [2]. Combined with the current situation of China's capital market, enterprises are affected by factors such as the initial conditions and the path of transition. The continuous changes in market and technology make enterprise investment activities face greater risks and uncertainties. Therefore, the analysis of the influencing factors of inefficient investment and how to improve investment efficiency are of great significance for the sustainable development of enterprises [3].

RETRACTED

It is a field of applied social psychology that studies the psychological activity rules of various people related to law. It is a borderline subject between law and psychology. It is playing an increasingly important role in the process of modernization of legal construction in China. The author makes a thorough elaboration on the psychological problems in illegal and criminal acts and judicial acts and further enriches and develops the application of the basic theories and technical methods of psychology in the judicial field. In practice, it contributes to the construction, reform, and improvement of the legal system.

## 2. Literature Review

Aiming at this research problem, Peng and Li expounded the theory of corporate governance, analyzed the advantages and realization ways of legal Psychology institutional investors in participating in corporate governance, and believed that legal Psychology institutional investors played the role of supervisor in corporate governance, which could improve corporate governance and reduce the degree of earnings management of the company to a certain extent [4]. Setiawati et al. studied the mechanism of institutional investors' participation in corporate governance. Whether institutional investors participate in corporate governance mainly depends on the comparison of the possible income of investment and the cost of investment. They analyzed the influencing factors of their participation in corporate governance from the inside and outside and considered the investment style of institutional investors. They believe that securities prefer companies with short-term returns and their investment operations are frequent, while social security funds prefer companies with less risk. They have high enthusiasm to participate in corporate governance and pursue long-term interests [5]. Viviers and Mans-Kemp explored its impact on the performance of corporate governance from the perspective of institutional investors through empirical means. They all concluded that the existence of institutional investors can effectively improve the company's performance [6]. Rey et al. believed that the performance of listed companies with institutional investors is significantly higher than that without institutional investors, and the information disclosure level of listed companies with institutional investors is also significantly higher than that without institutional investors [7]. Anoshkina et al. believed that the disclosure level of companies with institutional investors is also significantly higher than that of companies without institutional investors [8]. Tran and Pham believed that different investment strategies of institutional investors also have different effects on corporate performance [9]. Andryeyeva et al. believed that only institutional investors such as pension funds can play a greater role in corporate governance, and mutual funds and insurance companies do not play an active role. In the financial system, restrictions on the shareholding ratio and voting rights of institutional investors will affect their enthusiasm to participate in corporate governance [10]. Nurazi et al. believed that the heterogeneity of institutional investors has different effects on corporate governance. Pressure-sensitive institutional investors have a negative correlation with corporate performance and have no significant relationship with executive compensation [11]. Siddiqui and Singh tested the correlation between institutional investors and corporate social responsibility through a panel data model and reached the following conclusions: institutional investors' shareholding is significantly positively correlated with the contribution rate of government income and social income, and institutional investors prefer to invest in companies that undertake government and social responsibility [12]. Qi and Cheng pointed out that the field research of institutional investors has a governance effect on enterprise information disclosure, which helps to improve the quality of information disclosure. In addition, the field research of institutional investors may also encourage the management to predict earnings in a fuzzy way, increase insider transactions, curb excessive investment, and promote enterprise innovation [13].

RETRACTED

Based on the current research, the research conclusion of this article has positive policy significance. The first is to give full play to the role of field research of institutional investors in promoting enterprise environmental governance. Therefore, institutional investors should be actively encouraged to conduct field research on heavily polluting enterprises and ask targeted questions. The media and local environmental protection departments can participate at the same time. The second is to fundamentally reduce the degree of environmental information asymmetry. This study shows that access to environmental information helps stakeholders to supervise corporate environmental governance. Therefore, we should formulate and issue policies and regulations that require enterprises to disclose environmental information as soon as possible, improve the standards of environmental information disclosure, establish an enterprise environmental information disclosure platform, and improve the level and quality of environmental information disclosure.

## 3. Methods

### 3.1. Assumptions

At present, there are no standardized disclosure requirements for environmental information of enterprises by regulatory authorities, which increases the asymmetry of environmental information, weakens the external supervision of enterprise environmental governance, and leads to the lack of motivation of enterprise environmental governance. Institutional investors understand the operation status of enterprises through factory visits and on-site inquiries, which provides a unique situation for reducing information asymmetry. After the field investigation, institutional investors need to disclose the investigation to the public through the investor relations activity record form. Information disclosure can introduce external supervision, so as to promote the environmental governance of enterprises [14].

First, when the field investigation reveals the environmental information of enterprises, investors in the market can punish and play a supervisory role by “voting with their feet” for enterprises with poor environmental governance. Based on the above analysis, this article puts forward the research Hypothesis 1.

**Hypothesis 1 .**

The field research of institutional investors can promote the environmental governance of enterprises.

Institutional investors conduct field research to alleviate environmental information asymmetry and urge enterprises to actively carry out environmental governance. However, the environmental information disclosure status and operating characteristics of different enterprises are different, and the mitigation degree of environmental information asymmetry by field research is also different, which ultimately affects the governance effect of investors' field research.

On the one hand, for enterprises with better information disclosure, investors can timely understand the operation status of the company according to the information released by the enterprise, and the incremental information obtained from field research is limited. For enterprises with poor environmental information disclosure, institutional investors can collect more environmental information through field research, alleviate environmental information asymmetry, and play a relatively stronger role in environmental governance [15]. On the other hand, listed companies generally have more and widely distributed subsidiaries, which are the main units causing environmental pollution. According to statistics, more than 90% of the research occurred in the location of the enterprise headquarters. If the distribution of parent companies and subsidiaries is relatively concentrated, institutional investors collect more environmental information in the field investigation process, alleviate the asymmetry of environmental information, and play a more obvious role in the effect of enterprise environmental governance [16, 17]. Based on the above analysis, this article puts forward research Hypothesis 2 and Hypothesis 3.

RETRACTED

**Hypothesis 2 .**

For enterprises with poor environmental information disclosure, the impact of field research of legal Psychology institutional investors on enterprise environmental governance is more obvious.

**Hypothesis 3 .**

For enterprises with more concentrated distribution, the impact of field research of legal Psychology institutional investors on enterprise environmental governance is more obvious.

As a kind of legal or institutionalized power, leadership power is the result of the development and evolution of human society. It is to maintain and strengthen the cooperation of human society, reduce the cost of interpersonal interaction, and promote the realization of the overall and collective interests of society. In essence, it is a relationship between legal system and class social interests. Leadership power is a comprehensive and systematic project with three attributes of management science, social psychology, and law, and its essence is the socialization of legal psychology.

### 3.2. Sample Selection

This article takes the listed companies in the A-share heavy pollution industry of Shenzhen Stock Exchange from 2018 to 2021 as the initial research sample, excludes ST *∗* ST companies and samples with missing values, and finally obtains 2246 observations. It includes 8 industries: Food and beverage industry; hydropower and gas industry; papermaking and printing industry; petrochemical and plastic industry; biomedical industry; metal and nonmetal industry; textile, clothing, leather, and wool industry; and mining industry [18]. In order to eliminate the influence of outliers on the research conclusions, all continuous variables are reduced by 1% and 99% quantiles. The data on environmental protection investment and pollutant discharge fee of enterprises are obtained by manually collecting the annual reports of listed companies. Other data are from the wind database and CSMAR database. Stata13.0 is used to process and analyze the data [19].

In this article, the cumulative number of on-site investigations of enterprises in the current year + 1 is used as the measurement index of on-site investigations of legal Psychology institutional investors, which is expressed by Investigate. In the robustness test part, the virtual variables are set by whether the enterprise is investigated in the field in that year.

RETRACTED

### 3.3. Environmental Information Disclosure and Enterprise Distribution Concentration

Corporate environmental information disclosure indicators are measured by Runling global rating (RKS). The RKS score is issued annually by Runling Global Consulting Co., Ltd., an independent third-party rating agency, to score the environmental information related to the total annual investment in environmental protection transformation and annual carbon emission reduction of enterprises in the social responsibility report of listed companies, with a full score of 100. The Runling global rating score can effectively distinguish the degree of environmental information disclosure of enterprises. In this article, the original score is divided by 100 and is expressed by Score [20]. Using the distribution of subsidiaries and parent companies to measure, the index construction process is as follows: first, eliminate the subsidiaries with a shareholding ratio of less than 50% of the parent company, exclude the overseas registered subsidiaries, then manually search the registration place of subsidiaries and match with the parent company, and finally calculate the proportion of subsidiaries distributed in the same province of the same parent company, expressed by Comprov.

### 3.4. Control Variables

Considering that there are many factors affecting corporate environmental governance, the control variables of this article are selected from three levels: enterprise, region, and manager characteristics. The indicators at the enterprise level include financial leverage (Lev), company size, growth, profitability (ROE), company age (age), property right nature (SOE), market competitiveness (HHI), and shareholding ratio of institutional investors (Inst). Factors at the regional level include the regional legal environment and legal system (index), regional investment in environmental pollution control (invest), and the number of people in regional environmental law enforcement (people). Factors at the level of manager characteristics include age, gender, and education of managers. See Tables 1 and 2 for detailed definitions of variables.

### 3.5. Model Design

This article uses the following model to test the impact of field research by institutional investors on corporate environmental governance:

(1) $$\begin{array}{c} Env_{i,t}=\alpha_{0}+\alpha_{1}{\text{Investigate}}_{i,t}+\text{Ctrls}+\text{Year}+\text{Industry}+\varepsilon_{i,t}, \end{array}$$

(2) $$\begin{array}{c} Env_{i,t}=\beta_{0}+\beta_{1}{\text{Investigate}}_{i,t}\times X_{i,t}+\text{Ctrls}+\text{Year}+\text{Industry}+\varepsilon_{i,t}, \end{array}$$

where *Env*_*i*,*t*_ represents the environmental governance of the enterprise. The main inspection part is measured by the environmental protection investment of the enterprise, and the robustness inspection part is replaced by the sewage charge. Investigate_*i*,*t*_ is the main explanatory variable of this article, indicating the field research of institutional investors [21, 22]. In equation (2), *X* represents the indicators of enterprise environmental information disclosure (Score) and enterprise distribution concentration (Compror). According to the research hypothesis of this article, *α*_1_ in formula (1) is significant and *β*_3_ in formula (2) is significant.

RETRACTED

### 3.6. Multiple Linear Regression Model

A multiple regression model is established for the empirical test. Among them, UNRD is the explanatory variable, indicating the degree of insufficient innovation investment; *INS*_*Y*_ and *INS*_*H*_ are explanatory variables to measure whether institutional investors hold shares and the overall shareholding ratio of institutional investors in companies with institutional investors. At the same time, in the model, we control the company size, profitability, growth capacity, investment opportunities, solvency, equity concentration, shareholding ratio of senior executives, size of the board of directors, proportion of independent directors, industry, and year to avoid its impact on the empirical results [23, 24]. The multiple regression model is as follows:

(3) $$\begin{array}{c} \beta_{0}+\beta_{1}INS_{Yi,t}+\beta_{2}SIZE_{i,t}+\beta_{3}HL\;D-5_{i,t}+\beta_{4}ROE_{i,t}+\beta_{5}BSIZE_{i,t}+\beta_{6}MGT_{i,t}+\beta_{7}IND_{i,t}+\beta_{8}LEV_{i,t}+\beta_{9}CSALE_{i,t}+\beta_{10}PB_{i,t}+YEAR+IN\;D+\varepsilon_{1}\\ UNR\;D=\beta_{0}+\beta_{1}INS_{Yi,t}+\beta_{2}SIZE_{i,t}+\beta_{3}HL\;D-5_{i,t}+\beta_{4}ROE_{i,t}+\beta_{5}BSIZE_{i,t}+\beta_{6}MGT_{i,t}+\beta_{7}IND_{i,t}+\beta_{8}LEV_{i,t}+\beta_{9}CSALE_{i,t}+\beta_{10}PB_{i,t}+YEAR+IN\;D+\varepsilon_{1}\\ \beta_{0}+\beta_{1}INS_{Hi,t}+\beta_{2}SIZE_{i,t}+\beta_{3}HL\;D-5_{i,t}+\beta_{4}ROE_{i,t}+\beta_{5}BSIZE_{i,t}+\beta_{6}MGT_{i,t}+\beta_{7}IND_{i,t}+\beta_{8}LEV_{i,t}+\beta_{9}CSALE_{i,t}+\beta_{10}PB_{i,t}+YEAR+IN\;D+\varepsilon_{1},\\ UNR\;D=\beta_{0}+\beta_{1}INS_{Hi,t}+\beta_{2}SIZE_{i,t}+\beta_{3}HL\;D-5_{i,t}+\beta_{4}ROE_{i,t}+\beta_{5}BSIZE_{i,t}+\beta_{6}MGT_{i,t}+\beta_{7}IND_{i,t}+\beta_{8}LEV_{i,t}+\beta_{9}CSALE_{i,t}+\beta_{10}PB_{i,t}+YEAR+IN\;D+\varepsilon_{1}\\ \beta_{0}+\beta_{1}INS_{Ri,t}+\beta_{2}INS_{Mi,t}+\beta_{3}SIZE_{i,t}+\beta_{4}HL\;D-5_{i,t}+\beta_{5}ROE_{i,t}+\beta_{6}BSIZE_{i,t}+\beta_{7}MGT_{i,t}+\beta_{8}IND_{i,t}+\beta_{9}LEV_{i,t}+\beta_{10}CSALE_{i,t}+\beta_{11}PB_{i,t}+YEAR+IN\;D+\varepsilon_{1},\\ UNR\;D=\beta_{0}+\beta_{1}INS_{Ri,t}+\beta_{2}INS_{Mi,t}+\beta_{3}SIZE_{i,t}+\beta_{4}HL\;D-5_{i,t}+\beta_{5}ROE_{i,t}+\beta_{6}BSIZE_{i,t}+\beta_{7}MGT_{i,t}+\beta_{8}IND_{i,t}+\beta_{9}LEV_{i,t}+\beta_{10}CSALE_{i,t}+\beta_{11}PB_{i,t}+YEAR+IN\;D+\varepsilon_{1}\\ \beta_{0}+\beta_{1}STABLE_{i,t}+\beta_{2}SIZE_{i,t}+\beta_{3}HL\;D-5_{i,t}+\beta_{4}ROE_{i,t}+\beta_{5}BSIZE_{i,t}+\beta_{6}MGT_{i,t}+\beta_{7}IND_{i,t}+\beta_{8}LEV_{i,t}+\beta_{9}CSALE_{i,t}+\beta_{10}PB_{i,t}+YEAR+IN\;D+\varepsilon_{1},\\ UNR\;D=\beta_{0}+\beta_{1}STABLE_{i,t}+\beta_{2}SIZE_{i,t}+\beta_{3}HL\;D-5_{i,t}+\beta_{4}ROE_{i,t}+\beta_{5}BSIZE_{i,t}+\beta_{6}MGT_{i,t}+\beta_{7}IND_{i,t}+\beta_{8}LEV_{i,t}+\beta_{9}CSALE_{i,t}+\beta_{10}PB_{i,t}+YEAR+IN\;D+\varepsilon_{1}\\ \beta_{0}+\beta_{1}INS_{Yi,t}+\beta_{2}INS_{Yi,t}*AREA_{i,t}+\beta_{3}AREA_{i,t}+\beta_{4}SIZE_{i,t}+\beta_{5}HL\;D-5_{i,t}+\beta_{6}ROE_{i,t}+\beta_{7}BSIZE_{i,t}+\beta_{8}MGT_{i,t}+\beta_{9}IND_{i,t}+\beta_{10}LEV_{i,t}+\beta_{11}CSALE_{i,t}+\beta_{12}PB_{i,t}+YEAR+IN\;D+\varepsilon_{1},\\ UNR\;D=\beta_{0}+\beta_{1}INS_{Yi,t}+\beta_{2}INS_{Yi,t}*AREA_{i,t}+\beta_{3}AREA_{i,t}+\beta_{4}SIZE_{i,t}+\beta_{5}HL\;D-5_{i,t}+\beta_{6}ROE_{i,t}+\beta_{7}BSIZE_{i,t}+\beta_{8}MGT_{i,t}+\beta_{9}IND_{i,t}+\beta_{10}LEV_{i,t}+\beta_{11}CSALE_{i,t}+\beta_{12}PB_{i,t}+YEAR+IN\;D+\varepsilon_{1}\\ \beta_{0}+\beta_{1}INS_{Hi,t}+\beta_{2}INS_{Hi,t}*AREA_{i,t}+\beta_{3}AREA_{i,t}+\beta_{4}SIZE_{i,t}+\beta_{5}HL\;D-5_{i,t}+\beta_{6}ROE_{i,t}+\beta_{7}BSIZE_{i,t}+\beta_{8}MGT_{i,t}+\beta_{9}IND_{i,t}+\beta_{10}LEV_{i,t}+\beta_{11}CSALE_{i,t}+\beta_{12}PB_{i,t}+YEAR+IN\;D+\varepsilon_{1},\\ UNR\;D=\beta_{0}+\beta_{1}INS_{Hi,t}+\beta_{2}INS_{Hi,t}*AREA_{i,t}+\beta_{3}AREA_{i,t}+\beta_{4}SIZE_{i,t}+\beta_{5}HL\;D-5_{i,t}+\beta_{6}ROE_{i,t}+\beta_{7}BSIZE_{i,t}+\beta_{8}MGT_{i,t}+\beta_{9}IND_{i,t}+\beta_{10}LEV_{i,t}+\beta_{11}CSALE_{i,t}+\beta_{12}PB_{i,t}+YEAR+IN\;D+\varepsilon_{1}\\ \beta_{0}+\beta_{1}INS_{Yi,t}+\beta_{2}INS_{Yi,t}*STATE_{i,t}+\beta_{3}STATE_{i,t}+\beta_{4}SIZE_{i,t}+\beta_{5}HL\;D-5_{i,t}+\beta_{6}ROE_{i,t}+\beta_{7}BSIZE_{i,t}+\beta_{8}MGT_{i,t}+\beta_{9}IND_{i,t}+\beta_{10}LEV_{i,t}+\beta_{11}CSALE_{i,t}+\beta_{12}PB_{i,t}+YEAR+IN\;D+\varepsilon_{1},\\ UNR\;D=\beta_{0}+\beta_{1}INS_{Yi,t}+\beta_{2}INS_{Yi,t}*STATE_{i,t}+\beta_{3}STATE_{i,t}+\beta_{4}SIZE_{i,t}+\beta_{5}HL\;D-5_{i,t}+\beta_{6}ROE_{i,t}+\beta_{7}BSIZE_{i,t}+\beta_{8}MGT_{i,t}+\beta_{9}IND_{i,t}+\beta_{10}LEV_{i,t}+\beta_{11}CSALE_{i,t}+\beta_{12}PB_{i,t}+YEAR+IN\;D+\varepsilon_{1}\\ \beta_{0}+\beta_{1}INS_{Hi,t}+\beta_{2}INS_{Hi,t}*STATE_{i,t}+\beta_{3}STATE_{i,t}+\beta_{4}SIZE_{i,t}+\beta_{5}HL\;D-5_{i,t}+\beta_{6}ROE_{i,t}+\beta_{7}BSIZE_{i,t}+\beta_{8}MGT_{i,t}+\beta_{9}IND_{i,t}+\beta_{10}LEV_{i,t}+\beta_{11}CSALE_{i,t}+\beta_{12}PB_{i,t}+YEAR+IN\;D+\varepsilon_{1},\\ UNR\;D=\beta_{0}+\beta_{1}INS_{Hi,t}+\beta_{2}INS_{Hi,t}*STATE_{i,t}+\beta_{3}STATE_{i,t}+\beta_{4}SIZE_{i,t}+\beta_{5}HL\;D-5_{i,t}+\beta_{6}ROE_{i,t}+\beta_{7}BSIZE_{i,t}+\beta_{8}MGT_{i,t}+\beta_{9}IND_{i,t}+\beta_{10}LEV_{i,t}+\beta_{11}CSALE_{i,t}+\beta_{12}PB_{i,t}+YEAR+IN\;D+\varepsilon_{1}, \end{array}$$

RETRACTED

## 4. Results and Analysis

### 4.1. Descriptive Statistics

Tables 3 and 4 show the descriptive statistical results of the main variables in this article. It can be seen that the average value of the enterprise environmental governance indicators standardized with the total assets of the enterprise is 0.404 and the median is 0. The average value of enterprise environmental governance indicators standardized with total enterprise income is 0.978, and the maximum and minimum values are 20.255 and 0, respectively. The average value of the sample of institutional investor field survey is 1.133 and the median is 1.098. It can be seen that the deviation degree of the sample is small, and the maximum and minimum values are 3.179 and 0, respectively, indicating that there are certain differences between the samples. The average value of environmental information disclosure (Score) is 0.079 and the maximum value is 0.586. Generally speaking, the environmental information disclosure is not good. The average value of enterprise distribution concentration index (Comprov) is 0.577, indicating that the distribution of parent companies and subsidiaries is at a moderate level [25]. Among other control variables, the mean value of asset liability ratio (Lev) is 0.393, the mean value of growth is 0.099, and the mean value of property right (Soe) is 0.272, which are consistent with existing studies.

### 4.2. Univariate Test

In order to more intuitively investigate the relationship between the field research of institutional investors and corporate environmental governance, this article groups enterprises according to whether they are investigated by institutional investors and compares the differences between the environmental capital investment of the two groups.  Table 5 and Figure 2 report the results of univariate analysis. It can be seen from the table that the average value of the environmental governance indicators of the investigated enterprises is 0.431, which is higher than the average value of the samples that have not been investigated by 0.338. Through *t*-test, the results remain significant at the level of 10%. The average value of enterprise environmental governance indicators is 1.047, which is greater than 0.821 of enterprises that have not been investigated. The results of *t*-test are significant at the level of 10%. The above results show that the enterprises surveyed by institutional investors have high environmental capital investment, which preliminarily verifies the previous Hypothesis 1. In this article, the investigated enterprises are further grouped according to the average value of environmental information disclosure and company distribution concentration (see Tables 6 and 7 and Figures 3 and 4). If the enterprise information disclosure level (Score) is higher than the average value (0.079), it is considered that the environmental information disclosure is good; on the contrary, the environmental information disclosure is poor. If the enterprise distribution concentration (Compror) is higher than the average (0.577), it is considered that the enterprise distribution is more concentrated; on the contrary, the distribution is more scattered. The test results are shown in Tables 6 and 7 and Figures 3 and 4. It can be seen that among the surveyed enterprises, the environmental capital investment of enterprises with poor environmental information disclosure (0.479 and 1.161) is higher than that of enterprises with good environmental information disclosure (0.252 and 0.618). The mean *t*-test maintains the significance level of 1%, indicating that the impact of field research on enterprise environmental governance is more obvious in enterprises with poor environmental information disclosure, which preliminarily verifies Hypothesis 2 of this article. Similarly, when the enterprise distribution is more concentrated, the enterprise environmental capital investment is 0.536 and 1.286, which is higher than the enterprise environmental capital investment with more scattered distribution (0.315 and 0.778) and maintains the significance level of 1%, which preliminarily verifies the Hypothesis 3 of this article. Univariate analysis has preliminarily verified the above assumptions and the following will be further tested by regression analysis.

RETRACTED

### 4.3. Regression Analysis

In order to further investigate the impact of field research of institutional investors on corporate environmental governance, this article makes a regression test on equation (1), and the results are listed in Tables 8 and 9. It can be seen from the tables that in uncontrolled years and industries, the regression coefficients of institutional investor investigation and enterprise environmental protection capital investment are 0.0703 and 0.2416, respectively, which are significant at the level of 5%. After controlling the year and industry, the regression results show that the field investigation of institutional investors and enterprise environmental capital investment are still positive, significantly at the level of 5% and 1%, respectively. That is, the field research of institutional investors is helpful to promote the environmental governance of enterprises.

### 4.4. Further Inspection

The results of further tests are shown in Tables 10–13. It can be seen from Tables 10 and 11 that the coefficient of the investigate × score is negative and significant at the level of 5%. This result has not changed significantly after the control year and industry, indicating that for enterprises with poor quality of environmental information disclosure, the impact of field research by institutional investors on their environmental governance is more obvious, which supports Hypothesis 2. It can be seen from Tables 12 and 13 that the coefficients of the investigate × complex are positive, which are significant at the level of 5%, and the results have not changed significantly after controlling the year and industry, which verifies Hypothesis 3. The above research results show that the environmental disclosure of subsidiaries has a more obvious impact on the local investors. For enterprises with worse quality of environmental information and more concentrated distribution of subsidiaries, more environmental information is obtained through field research, the degree of environmental information asymmetry is reduced, and the effect of environmental governance is more obvious.

### 4.5. Robustness Test

In order to further verify the reliability of the conclusion of this article, considering the possible problems in endogeneity, model setting, and index measurement, this article adopts the following methods to re-estimate the model: First, the two-stage least square method is used to estimate whether the parent company's headquarters is located in the prefecture level city in that year and whether there are high-speed railways and airports and flights. Second, the propensity score matching method is used for 1 : 1 sample matching to eliminate the differences between samples, and the matched samples are used to re-estimate. Third, the Tobit model is used to re-estimate. Fourth, the logarithmic environmental capital investment is taken as the index of environmental governance, and the level of environmental governance is measured by dividing the sewage charge by the total assets. Fifth, the enterprise is investigated and set up virtual variables is used as the measurement index of field investigation of institutional investors.

RETRACTED

#### 4.5.1. Standardizing Leadership Power with the Legal System

To regulate the leading power, we must first regulate and control its power resources legally and establish a legal system for regulating the operation of leading power. The restrictive relationship of leading power is essentially a problem of leading power structure, so the regulation of leading power must start from the leading power structure. One is to strictly distinguish the two different levels of leadership power structure and leadership power operation. The other is to explore the new mechanism of leadership power checks and balances under the decentralization system and leadership power checks and balances under the centralized system. Three principles should be adhered to standardize the leadership power with the legal system: first, the allocation and exercise of leadership power should comply with the constitutional and legal principles; second, the allocation and exercise of leadership power should comply with the principle of respecting rights; and third, the allocation and exercise of leadership power should comply with the principle of the unity of power and responsibility. The psychological mechanism of leadership power has the characteristics of indeterminacy, double-edged, mandatory, intersubjectivity, and usefulness. One is uncertainty. The exercise of leading power is based on the free will of the power subject, which determines that leading power has the characteristics of uncertainty in content and reality transformation. The second is double-edged. The duality of leading power is good or evil, good or bad, and it also affects the destiny of the power holder and the public interests of the society. Third, it is mandatory. Coercive force is the concentrated embodiment of the characteristics of leading power, which in essence imposes the will of the leader on the conscious behavior of others. Fourth, intersubjectivity. The intersubjectivity of psychological mechanism of leading power includes the individuality of belonging relation and the intersubjectivity of operating field. Fifth, utility. The alienation form of power rent-seeking exists in the exercise of leading power. When analyzing Chinese society in the sociocultural context, it belongs to the rational society in essence, and the network of organizational relations is an important social form.

## 5. Conclusion

This article studies the impact of legal Psychology institutional investors on corporate governance environment. From 2018 to 2021, taking the highly polluting listed companies of Shenzhen Stock Exchange as the research sample, the impact of legal Psychology institutional investors on environmental governance and its mechanism is analyzed. The research shows that the field research of legal Psychology institutional investors plays a positive role in supporting enterprise environmental governance, while the field research of legal Psychology institutional investors plays a more important role in environmental governance for enterprises with incomplete environmental information and enterprises with more local subsidiaries. Further research on the impact of field research companies on environmental governance found that the field research of legal Psychology institutional investors supports stock market supervision and media supervision on corporate environmental governance. This study confirms the role of information inequality theory in environmental governance, expands the research scope of economic significance of field research, and has important practical significance for deepening understanding and promoting China's environmental governance. Follow-up researchers can extend the time span to enhance the reliability of data conclusions. At present, the methods of measuring environmental uncertainty are not consistent. Social distance makes it easy for leaders to stereotype or prejudice others, while activating the approach system will make leaders pay more attention to the reward target and underestimate or ignore the existence of risks. Control illusion often makes leaders overestimate their own value and abilities and lead to decision-making mistakes. From the perspective of external characteristics, the psychological mechanism of leadership power has the characteristics of uncertainty, double-edged, compulsion, intersubjectivity, use, and benefit, which implies the conditions for the expansion of leadership power and the abuse of leadership power. The accurate estimation of environmental uncertainty is very important for relevant research. We need to consider the characteristics of China's capital market and improve the estimation model in order to make the empirical results more convincing.

RETRACTED

## Figures and Tables

**Figure 1:** Industrial chain of private equity investment.

**Figure 2:** Univariate analysis chart (grouped by whether it is grouped by investigation).

**Figure 3:** Univariate analysis chart (grouped by the degree of environmental information disclosure).

**Figure 4:** Univariate analysis chart (grouped by the distribution of subsidiaries).

**Table 1:** Definition of relevant variables (1).

Variable name	Variable definition
*Env*_1_	Environmental protection investment divided by total assets × 100
*Env*_2_	Environmental protection investment divided by operating income × 100
Investigate	The number of times investigated in the year + 1 is taken as the logarithm
Score	Runling global rating (RKS) score divided by 100
Comprov	Calculate the proportion of subsidiaries of the same parent company in the same province
Lev	Asset liability ratio
Growth	Growth rate of operating revenue
Size	Total number of enterprises at the end of the year + 1 takes logarithm
Soe	Property right nature: 1 for state-owned enterprises, and 0 for vice versa
Roe	Return on net assets
Age	The logarithm of the company's founding age + 1

**Table 2:** Definition of relevant variables (2).

Variable name	Variable definition
HHI	Herfindal index
Inst	Shareholding ratio of institutional investors
Index	Market index
Inest	The total investment of provincial environmental pollution control is taken as logarithm
People	The total number of personnel in the provincial environmental protection system is taken as logarithm
Dage	Chairman's age divided by 100
Gender	If the gender of the chairman is male, the value is 1, otherwise it is 0
Education	Educational background of the chairman, 1 = technical secondary school or below, 2 = college, 3 = bachelor, 4 = master
Year	Annual dummy variable
Industry	Industry dummy variable

**Table 3:** Descriptive statistical analysis of main variables (1).

Variable	Number of samples	Mean value	Variance	Median	Minimum value	Maximum
*Env*_1_	2246	0.404	1.029	0	0	6.192
*Env*_2_	2246	0.978	2.883	0	0	20.255
Investigate	2246	1.133	0.936	1.098	0	3.179
Score	2246	0.079	0.166	0	0	0.586
Comprov	2088	0.577	0.321	0.601	0	1
Lev	2246	0.393	0.211	0.369	0.038	0.924
Growth	2246	0.099	0.274	0.071	−0.544	1.171
Size	2246	7.588	1.076	7.514	5.018	10.584
Soe	2246	0.272	0.445	0	0	1

**Table 4:** Descriptive statistical analysis of main variables (2).

Variable	Number of samples	Mean value	Variance	Median	Minimum value	Maximum
Roe	2246	0.053	0.137	0.063	−0.667	0.321
Age	2246	2.873	0.258	2.891	2.198	3.527
HHI	2246	0.084	0.078	0.064	0.018	0.414
Inst	2246	0.379	0.233	0.388	0.006	0.857
Index	2246	7.749	1.794	7.931	2.531	9.881
Invest	2246	5.834	0.704	5.849	3.101	6.858
People	2246	8.963	0.658	9.165	6.848	10.205
Dage	2246	0.533	0.072	0.531	0.361	0.711
Gender	2246	0.956	0.209	1	0	1
Education	2246	3.079	1.316	3	0	5

**Table 5:** Univariate analysis to determine whether it is grouped by investigation.

Variables	Visit = 0		Visit = 1		Mean-diff
	*N*	Mean	*N*	Mean	
*Env*_1_	669	0.338	1577	0.431	−0.092
*Env*_2_	669	0.821	1577	1.047	−0.227

**Table 6:** Univariate analysis (grouped by the degree of environmental information disclosure).

Variables	Score > mean		Score < mean		Mean-diff
	*N*	Mean	*N*	Mean	
*Env*_1_	332	0.252	1245	0.479	−0.228
*Env*_2_	332	0.618	1245	1.161	−0.542

RETRACTED

**Table 7:** Univariate analysis (grouped by the distribution of subsidiaries).

Variables	Comprov < mean		Comprov > mean		Mean-diff
	N	Mean	N	Mean	
*Env*_1_	746	0.315	831	0.536	−0.222
*Env*_2_	746	0.778	831	1.286	−0.507

**Table 8:** Field research of institutional investors and corporate environmental governance (1).

	(1)	(2)	(3)	(4)
	*Env*_1_	*Env*_1_	*Env*_2_	*Env*_2_
Investigate	0.0703	0.0783	0.2416	0.2787
Lev	0.5282	0.3241	1.6656	0.8978
Growth	−0.1011	−0.0856	−0.2414	−0.1787
Size	−0.0432	0.0025	−0.2419	−0.0673
Soe	0.1974	0.1012	0.5785	0.2105
Roe	0.4264	0.1442	0.7002	−0.3645
Age	−0.2008	−0.2838	−0.1643	−0.5143
HHI	−0.5623	−0.8088	−1.5489	−2.7064

**Table 9:** Field research of institutional investors and corporate environmental governance (2).

	(1)	(2)	(3)	(4)
	*Env*_1_	*Env*_1_	*Env*_2_	*Env*_2_
Inst	0.0449	−0.0228	0.2028	−0.0592
Index	−0.0288	−0.0276	−0.0918	−0.0858
Invest	−0.0086	−0.0185	−0.1862	−0.2243
People	0.0774	0.0847	0.1421	0.1719
Dage	−0.3005	−0.3379	−0.4035	−0.5549
Gender	−0.0596	−0.0437	−0.5074	−0.4621
Education	−0.0101	−0.0126	−0.0724	−0.0831
_Cons	0.8125	0.8964	3.6865	4.2158

**Table 10:** Field research of institutional investors and corporate environmental governance (test results of environmental information disclosure) (1).

	(1)	(2)	(3)	(4)
	*Env*_1_	*Env*_1_	*Env*_2_	*Env*_2_
Investigate	0.1103	0.1202	0.3501	0.3939
Score	0.0627	0.0579	0.6881	0.6755
Investigate × score	−0.3816	−0.3967	−1.1274	−1.1868
Lev	0.5053	0.2985	1.6404	0.8619
Growth	−0.1166	−0.1029	−0.2771	−0.2203
Size	−0.0233	0.0238	−0.2078	−0.0281
Soe	0.2038	0.1076	0.5838	0.2165
Roe	0.4313	0.1461	0.7281	−0.3436
Age	−0.1824	−0.2676	−0.1264	−0.4797
HHI	−0.5768	−0.8261	−1.6457	−2.7691

**Table 11:** Field research of institutional investors and corporate environmental governance (test results of environmental information disclosure) (2).

	(1)	(2)	(3)	(4)
	*Env*_1_	*Env*_1_	*Env*_2_	*Env*_2_
Inst	0.0428	−0.0252	0.1849	−0.0788
Index	−0.0282	−0.0266	−0.0893	−0.0839
Invest	−0.0141	−0.0248	−0.1968	−0.2357
People	0.0793	0.0869	0.1525	0.1818
Dage	−0.3205	−0.3587	−0.4772	−0.6326
Gender	−0.0599	−0.0441	−0.5039	−0.4577
Education	−0.0038	−0.0061	−0.062–18	−0.0713
_Cons	0.6114	0.6918	3.2445	3.7277

**Table 12:** Field research of institutional investors and corporate environmental governance (test results of the distribution of subsidiaries) (1).

	(1)	(2)	(3)	(4)
	*Env*_1_	*Env*_1_	*Env*_2_	*Env*_2_
Investigate	−0.0452	−0.0499	−0.0599	−0.0686
Score	0.0533	−0.0356	−0.0281	−0.3372
Investigate × score	0.2148	0.2428	0.5651	0.6635
Lev	0.5608	0.3305	0–1.7817	0.9138
Growth	−0.0834	−0.0759	−0.2144	−0.1739
Size	−0.0403	0.0097	−0.2381	−0.0474
Soe	0.1698	0.0698	0.5245	0.1393
Roe	0.4179	0.1042	0.6812	−0.5038
Age	−0.1838	−0.2797	−0.1486	−0.5397
HHI	−0.6344	−0.9225	−1.8094	−3.0193

RETRACTED

**Table 13:** Field survey of institutional investors and corporate environmental governance (test results of the distribution of subsidiaries) (2).

	(1)	(2)	(3)	(4)
	*Env*_1_	*Env*_1_	*Env*_2_	*Env*_2_
Inst	−0.0055	−0.0827	0.1488	−0.1514
Index	−0.0278	−0.0278	−0.0892	−0.0897
Invest	0.0084	0.0033	−0.1438	−0.1599
People	0.0458	0.0571	0.0549	0.0962
Dage	−0.3215	−0.3536	−0.4194	−0.5382
Gender	−0.0769	−0.0526	−0.4735	−0.3925
Education	−0.0056	−0.0068	−0.0706	−0.0755
_Cons	0.9188	1.091	4.1209	4.6983

## Data Availability

The labeled data set used to support the findings of this study is available from the author upon request.
